The article "A Sensor-Based IoT Data Collection and Marine Economy Collaborative Innovation Method" was retracted in 2023. Reasons: unreliable results or conclusions; concerns about the data; concerns about the peer review; concerns about the citations.

# A Sensor-Based IoT Data Collection and Marine Economy Collaborative Innovation Method

**DOI:** 10.1155/2022/3421999

**Published:** 2022-03-15

**Authors:** Tao Liu, Fan Wu

**Affiliations:** ^1^College of Economics & Management, Shandong University of Science and Technology, Qingdao 266000, China; ^2^Shandong Academy of Social Sciences, Jinan 250000, China

## Abstract

Traditional marine pastures have made great contributions to human beings, but traditional marine pastures have also caused major harm to the marine natural environment. Modern technology represented by artificial intelligence has broad application prospects and significant potential and has the ability to innovate and enhance the conventional marine ranching business that is currently in recession. The particularity of China's marine ranching industry determines the combination of technologies such as underwater robots and the Internet of Things with the development of marine ranching to create a sustainable intelligent marine ranching industry in China. The growth of China's national economy is largely influenced by the development of the country's financial services industry. In order to better support the development of the real economy, it is necessary to establish a financial service system with controllable risks and complementary activities. This paper proposes to use the method of Internet of Things data collection combined with sensors to conduct economic analysis. By taking a number of data in recent years for research and analysis, the results show that financial service industry innovation has become an important part of improving the competitiveness of the industry and an important driving force for economic growth. The Internet of Things (IoT) business in China is a fast-growing industry with huge potential. From the perspective of international comparison, our country is currently in the early stage of the development of the Internet of Things, and a certain technology, industry, and application foundation has been established in the early stage of development. In the financial services business, the visual tracking provided by IoT technology has innovative potential. Introducing IoT technology into financial service business and identifying the driving force and process of financial innovation have practical significance for accelerating financial innovation.

## 1. Introduction

With the rapid development of economy and the continuous growth of population, the quality and quantity of food required by human beings are also improving. Therefore, marine resources and economy are playing a more and more important role in human survival and development.

The marine fishery in many marine areas has shown a gradual downward trend and is undergoing a severe test [1–5]. In particular, it is basically difficult for the Bohai Sea, one of the four sea areas, to form fishing news, and it has fallen into a very difficult situation. Since the 1990s, China's fishing capacity has gradually increased and increased sharply. The annual allowable limit fishing capacity of China's offshore waters is 8 million tons, which is far from meeting the demand. At present, the number of economic fish once rich in production, such as *Penaeus chinensis*, *Pseudosciaena crocea*, and hairtail, has decreased sharply and is difficult to catch. The seaweed fields in the northern sea area of China are gradually decreasing or even disappearing, and some large seaweed fields are also declining. Seaweed field plays a very important role. Its decline directly leads to the decline of the quality and quantity of fish and shellfish. A large amount of garbage in the ocean covers some sea areas, resulting in the current situation of marine desertification, which seriously reduces the quality and quantity of marine biological species, just like the phenomenon of land desertification [6]. At present, it has been difficult for marine biological resources to meet the needs of traditional marine fishing and mariculture.

The article "A Sensor-Based IoT Data Collection and Marine Economy Collaborative Innovation Method" was retracted in 2023. Reasons: unreliable results or conclusions; concerns about the data; concerns about the peer review; concerns about the citations.

In recent decades, with the rapid development of fisheries, the global marine catch has continued to rise, thus masking the decline of fishery resources to a certain extent. At present, with the increasing market demand, declining coastal fishery resources, and improving fishing technology, the development of deep-sea fishery is gradually developing, but geographically, the expansion of deep sea has reached the maximum. The fishery economy has suffered great losses, and the number and intensity of fishermen are still rising. In fact, the continuous decline of fishery resources has greatly damaged the marine ecosystem and will produce serious economic and social problems.

In view of the current situation of marine resources, selecting a reasonable mode of production and operation is an important guarantee for the sustainable development of marine resources [7]. Similar to large-scale farming on land, marine ranching can play an important role. The rational management and scientific planning of marine pasture have many significant advantages, which have an important impact on the improvement of biodiversity and marine ecological environment. In addition, it can also encourage fishermen to change their industries, which can not only solve the employment problem of fishermen, but also better promote the development of marine fishery industry [8–10]. The effective management of marine pasture plays a very important role in extending the industrial chain.

The article "A Sensor-Based IoT Data Collection and Marine Economy Collaborative Innovation Method" was retracted in 2023. Reasons: unreliable results or conclusions; concerns about the data; concerns about the peer review; concerns about the citations.

As a main mode of production and advanced production mode of marine agriculture and animal husbandry, marine pasture has the characteristics of high efficiency, environmental protection, health, and energy saving. It is the crystallization of the integration and development of high and new technologies such as marine ecosystem, marine life, modern marine science and marine ecological environment, and modern information control engineering technology and production management. Therefore, marine pastures will promote the development of marine economy and other industrial economy and will occupy a larger proportion in the national economy.

The research contributions of the paper are as follows:

1. A collaborative innovation method of sensor-based IoT data acquisition and marine economy is proposed
2. Propose the establishment of a financial service system with controllable risks and complementary activities
3. Introducing IoT technology into financial service business and identifying the driving force and process of financial innovation has practical significance for accelerating financial innovation

## 2. Overview of the Technology and Industry of the Internet of Things

### 2.1. The Technology of Internet of Things

When defining the Internet of Things, Ashton [11–14], an associate professor at MIT, stated that it was “a network of objects that are connected to the Internet using radio frequency identification [RFID], electronic coding (EPC), and other technologies.” According to the International Telecommunication Union, the Internet of Things is defined as the connectivity of any time, any place, and any item with any other. It has three characteristics, which are as follows: comprehensive perception, the wide application of various perception technologies; dependable transmission, dependable information sharing and interaction between objects; intelligent processing, including the control of information in the Internet of Things; and reliable transmission, information sharing, and interaction between objects. As seen in Figure 1, the Internet of Things system is often separated into three-tier architecture, with the perception layer at the bottom, the network layer at the middle, and the application layer at the top:

1. *Perception Layer*. The perception layer is the basic layer and key link of the Internet of Things architecture. It is to establish the connection between the physical world and the information world. The sensing layer is used to collect and convert information to obtain the information and status of monitored items, equipment, and environment. It is usually composed of sensors or controllers and short-distance transmission networks.
2. *Network Layer*. The network layer is the middle layer of the structure, which is used to establish the connection between the perception layer and the application layer to realize the transmission and circulation of information in the Internet of Things system, including access unit and access network.
3. *Application Layer*. The application layer is the top layer of the Internet of Things architecture. The application layer mainly realizes data management and processing with the help of data fusion, big data analysis, cloud computing, and other technologies, analysis, processing, and decision-making, as well as realizing or completing the pending intelligent application and service tasks, so as to realize the recognition and perception between things, people and things, and things and people.

The article "A Sensor-Based IoT Data Collection and Marine Economy Collaborative Innovation Method" was retracted in 2023. Reasons: unreliable results or conclusions; concerns about the data; concerns about the peer review; concerns about the citations.

There are three common network topologies in the application of Internet of Things technology: star topology, tree topology, and mesh topology [15].

#### 2.1.1. Star Topology

The star topology, as shown in Figure 2, includes a coordinator node and several terminal nodes. Each terminal node can only communicate with the coordinator node, and the communication between two adjacent coordinator nodes also needs to be forwarded through the coordinator node. Star topology is the simplest of the three network structures, but it has poor flexibility [16]. All communication needs to be carried out through the central coordinator node. Therefore, it consumes a lot of energy for the coordinator node and has high requirements for the configuration of the coordinator [17].

#### 2.1.2. Tree Topology

The tree topology, as shown in Figure 3, includes a coordinator node, several routing nodes, and several terminal nodes. The coordinator node is connected with several routing nodes and terminal nodes, and the routing nodes of its child nodes can also continue to be connected with several routing nodes and terminal nodes, which are connected layer by layer to form a tree structure. In the tree topology, each node can only communicate with its parent and child nodes. Therefore, the transmission of information between nodes has only a unique routing channel, and the network flexibility is poor [18].

#### 2.1.3. Mesh Topology

The mesh topology, as shown in Figure 4, includes a coordinator node, several routing nodes, and several terminal nodes. The coordinator node is connected with several routing nodes and terminal nodes, and the routing nodes of its child nodes can also continue to be connected with several routing nodes and terminal nodes, which are connected layer by layer to form a mesh structure. Compared with tree topology, in mesh topology, routing nodes can communicate not only with their parent and child nodes, but also with their brother nodes. Therefore, the network has high flexibility, information can choose the optimal path for transmission, and a multihop ad hoc network can be formed [19].

The article "A Sensor-Based IoT Data Collection and Marine Economy Collaborative Innovation Method" was retracted in 2023. Reasons: unreliable results or conclusions; concerns about the data; concerns about the peer review; concerns about the citations.

### 2.2. The Industry of the Internet of Things

The notion of the Internet of Things may be traced back to similar research conducted at the Massachusetts Institute of Technology in 1999. After that, with the help of information sensing technology, network transmission technology, and artificial intelligence technology, the application scope of Internet of Things technology will continue to grow, eventually establishing a distinct sort of technology. Because different sections of study are focusing on different components of the Internet of Things, the definition of the specific notion of the Internet of Things varies as well. Nonetheless, the core concept of IoT is as follows: it is founded on information sensing technology and information transmission technology, it is characterized by information exchange and communication using specific protocols, and it is characterized by intelligent identification and management functions. The creation of an intelligent network is done by linking all of the items in the planet. It is necessary to distinguish between three architectures in the Internet of Things' fundamental system: the perception layer, the network layer, and the application layer, all of which are interconnected by the appropriate software, hardware, and network infrastructure.

The Internet of Things industry is a collection of production activities or activities that are closely connected to production activities that are based on the use of the Internet of Things technology. In accordance with the findings of the associated study, the Internet of Things industrial composition is classified into two categories: limited meaning and broad meaning. Within the context of the Internet of Things, the term “Internet of Things industry” refers to the industrial field that has been directly formed by the advancement of Internet of Things technology. Examples of such industries include research and development, design and manufacture of core sensing equipment for the Internet of Things, and the design and manufacture of network communication modules. Application software development, system integration, and a variety of other services are available. In a broader sense, the Internet of Things industry includes other infrastructure and human resources that are required for the development of the Internet of Things industry, as well as new parts of education, training, and other industries that have emerged as a result of the application of Internet of Things technology. For the purposes of this study, we will use the term “Internet of Things industry” in a wide meaning, which means that we will look at the influence of activities linked to the Internet of Things industry on regional economic growth in a broad sense.

The article "A Sensor-Based IoT Data Collection and Marine Economy Collaborative Innovation Method" was retracted in 2023. Reasons: unreliable results or conclusions; concerns about the data; concerns about the peer review; concerns about the citations.

The Internet of Things industry, as a significant new industrial type, possesses a number of distinguishing qualities, the first of which is its inventive nature. Moreover, by constructing the Internet of everything, it has fundamentally altered the relationship between human activities and the material world, altered human perceptions of the material world, and enabled the discovery and creation of novel methods and theories supported by a wealth of information. It has the advantages of application innovation and can, without a doubt, contribute to the development of productivity. For the second time, it exhibits the features of high permeability. Instead of being a distinct industrial type, the Internet of Things industry has a tight relationship with each of the original three sectors, and the lines between them are becoming increasingly blurred. The high degree of penetration of the Internet of Things industry in conventional industries has significantly enhanced the efficiency of connection between diverse economic activities, and the overall efficiency of economic operation has been constantly improved as a result of this improvement. In addition, it possesses external economic characteristics; namely, it is based on diversified node information, with each node information being applicable to a variety of related Internet of Things systems, allowing it to realize the information sharing and interaction of all things and fundamentally alter the mode of economic operation.

### 2.3. Combination Form of Internet of Things Industry and Traditional Industry

In recent years, the technical level of Internet of Things has been continuously improved, and the promotion efficiency of traditional industries has also been reflected in an all-round way. The combination form of Internet of Things industry and traditional industry is shown in Table 1.

Using technology from the Internet of Things, it has changed the way businesses work. It has combined the management of things and human management in each production link, and this has led to the continuous improvement of the overall level of intelligence in the industry. This means that it can provide better services to customers.

The Internet of Things industry is not only an important branch of the tertiary industry, but also closely related to various industries. The application of Internet of Things equipment to the existing production, operation, and management system in relevant production can form a network connection between the elements in the development of traditional industries in the form of network and more accurately grasp the operation characteristics of different industries through information perception and transmission, It can more accurately analyze the weak links of resource utilization in the operation of traditional industries and provide a more accurate basis for management decisions through intelligent analysis. At the same time, through the direct transmission of decision-making information of the Internet of Things, it can also solve the disadvantages of cumbersome system and great influence of human factors in the traditional management system, effectively improve the application level of decision-making, and promote the continuous development of relevant industries in the direction of intelligence.

The article "A Sensor-Based IoT Data Collection and Marine Economy Collaborative Innovation Method" was retracted in 2023. Reasons: unreliable results or conclusions; concerns about the data; concerns about the peer review; concerns about the citations.

On the theoretical level, with the deepening of relevant research, the level of public awareness of the development of the Internet of Things industry is also increasing. As a result, the drive animal network industry not only organically combines with traditional industries, but also provides diversified support for the change of regional economic development direction and development mode and plays a very obvious role in promoting regional economic development.

## 3. Energy Balance Data Transmission Algorithm for Ocean Monitoring Sensor Networks Based on Sparse Deployment

Like terrestrial wireless sensor networks, ocean monitoring sensor networks use battery power, so battery energy is an important factor restricting the long-term operation of sensor networks. For ocean sensor networks, the energy problem is more prominent. First, it is difficult to charge or replace the battery underwater. Second, due to the high cost of ocean monitoring sensor nodes, the balanced energy consumption of a single node is particularly important in sparse deployment. However, because the node data is usually collected to the base station node (sin*l*) before being transmitted to the observer, this centralized data transmission will inevitably lead to the unbalanced consumption of node energy in the network. This unbalanced energy consumption will lead to the decline of network reliability if it is light, and the whole network will be divided into multiple unconnected subnetworks if it is serious, which will greatly shorten the network lifetime.

We consider a sparsely deployed ocean monitoring sensor network: underwater mooring monitoring system. This system can collect real-time perception data of the whole water area for a long time. These real-time ocean data can enable us to better understand the ocean, so as to solve some globalization problems, such as natural disaster prediction and global warming.

The article "A Sensor-Based IoT Data Collection and Marine Economy Collaborative Innovation Method" was retracted in 2023. Reasons: unreliable results or conclusions; concerns about the data; concerns about the peer review; concerns about the citations.

The traditional mooring ocean monitoring system consists of the following parts: anchor, anchor rope, and sea buoy (surface sink node). The buoy is equipped with wireless communication equipment to transmit data to users in real time through satellite or shore base station. The underwater sensor is fixed on the anchor rope to measure the temperature, conductivity, salinity, pressure, and current velocity at different depths. These sensors at different depths need to periodically transmit the monitoring data to the surface buoy.

There are two main applications of ocean monitoring sensor networks: event-driven and periodic awareness. In this paper, periodic sensor networks are studied, in which the nodes will always monitor the network environment and send the found information to the collection nodes. This kind of mooring monitoring system is periodically perceived. In order to evaluate the lifetime of the network, we divide the time into rounds. For simplicity, let us assume that each node generates a packet in a round of time.

### 3.1. Energy Model of Underwater Acoustic Wave Propagation

In this part, we introduce the underwater acoustic wave propagation energy consumption models.

#### 3.1.1. Passive Sonar Formula

The formula for the lower side gives the SNR of the underwater signal at the receiver:

(1) $$\begin{array}{c} \text{SNR}=\text{SL}-\text{TL}-\text{NL}+\text{DI}\geq \text{DT}, \end{array}$$

where SL is the signal intensity at the sound source, TL is the signal transmission loss, NL is the noise intensity, DI is the sonar direction gain, and DT is the detection threshold value of the sonar. Equation (1) is defined in dBre *μ* Pa, where 1*μ* Pa=0.67 × 10^−18^watts/*m*^2^. The following refers to the dBre *μ* Pa with dB.

In shallow waters, the size of the noise is related to the movement of the ship, the size of the wind, biological noise, and undersea earthquakes. In this paper, we take an NL of 70 dB in shallow waters. The deep sea is calmer than the shallow sea, taking NL as 50 dB. DI and SNR are associated with the demodulator and hydroreader used, here taking the typical value DI=3 dB, SNR=20 dB, respectively.

#### 3.1.2. Transmission Loss

Sonic signals do not spread equally in the shallow and deep seas.

Shallow sea refers to water of less than 100 m. The transmission of acoustic signals in shallow seas is confined to cylinders composed of the sea and sea floor. The propagation loss in the shallow seas can be expressed as

(2) $$\begin{array}{c} \text{TL}=10\text{ log }d+\text{ad}\times 10^{-3}, \end{array}$$

where *d* is the distance between the sender and the receiver (in meters), *a* is the absorption coefficient (in dB/km), and TL is in dB.

The article "A Sensor-Based IoT Data Collection and Marine Economy Collaborative Innovation Method" was retracted in 2023. Reasons: unreliable results or conclusions; concerns about the data; concerns about the peer review; concerns about the citations.

In the deep sea, sound waves are mainly spherical diffusion, and the propagation loss is mainly caused by spherical diffusion and absorption loss, which can be expressed as

(3) $$\begin{array}{c} \text{TL}=20\text{ log }d+\text{ad}\times 10^{-3}. \end{array}$$

From equations (2) and (3), it can be seen that the propagation loss of sound waves in deep and shallow waters is mainly caused by distance related transmission attenuation and frequency related absorption loss.

When the frequency of absorption coefficient *a* is greater than several hundred Hertz, it can be expressed as the following formula:

(4) $$\begin{array}{c} a=\frac{0.1f^{2}}{1+f^{2}}+\frac{40f^{2}}{4100+f^{2}}+2.75*10^{-4}f^{2}+0.003, \end{array}$$

where the unit of *a* is dB/km, and the frequency *f* unit is kHz.

When the sound wave frequency is small, the calculation formula of *a* is as follows:

(5) $$\begin{array}{c} a=0.11\left(\frac{f^{2}}{1+f^{2}}\right)+0.011f^{2}+0.002. \end{array}$$

#### 3.1.3. Transmit Power

The sound source signal strength SL is related to the signal strength of the transmitted signal at 1 m away from the signal source, which can be expressed as

(6) $$\begin{array}{c} \text{SL}=10\;\log\left(\frac{I_{T}}{1\mu \text{ Pa}}\right). \end{array}$$

Among these, unit of *I*_*T*_ is *μ* Pa.

Using formula (6), you can get *I*_*T*_ as follows:

(7) $$\begin{array}{c} I_{T}=10^{\left(\text{SL}/10\right)}*0.67*10^{-18}, \end{array}$$

where *P*_*T*_(*d*) is in Watts/*m*^2^ and *H* is the depth of water in meters.

For deep sea, the transmission power of the source node shall be

(8) $$\begin{array}{c} P_{T}\left(d\right)=4\pi \times {\left(1m\right)}^{2}\times I_{T}. \end{array}$$

Using the above formula, we can calculate the transmission power required for signal transmission under a given transmission distance *d* and signal frequency *f*.

From equation (1), we get SL:

(9) $$\begin{array}{c} \text{SL}=\text{SNR}+\text{TL}+\text{NL}-\text{DI}, \end{array}$$

where the TL can be calculated by equations (2) and (3).

Then, by equation (7), it yields the signal intensity *I*_*T*_, and by formulas (8) and (9), the required emission power *P*_*T*_ is obtained.

For shallow seas, an emission power *P*_*T*_ can be obtained by the following equation:

(10) $$\begin{array}{c} P_{T}\left(d\right)=P_{T_{\text{shallow}}}\left(d\right)=2\pi H\times 10^{\left(\text{SL}/10\right)}\times 0.67\times 10^{-18}. \end{array}$$

For the deep sea, the transmission power *P*_*T*_ can be obtained as

(11) $$\begin{array}{c} P_{T}\left(d\right)=P_{T_{\text{deep}}}\left(d\right)=4\pi \times 10^{\left(\text{SL}/10\right)}\times 0.67\times 10^{-18}. \end{array}$$

The article "A Sensor-Based IoT Data Collection and Marine Economy Collaborative Innovation Method" was retracted in 2023. Reasons: unreliable results or conclusions; concerns about the data; concerns about the peer review; concerns about the citations.

### 3.2. The Reason for the Imbalance of Energy Consumption

In this part, we analyze the reasons for the imbalance of energy consumption caused by the network model. Underwater linear network structure is shown in Figure 5.

Suppose the underwater sensor node *S*={*S*_*i*_*|i* ∈ {1,…, *n*}} constitutes a chain sensor network, as shown in Figure 5. To facilitate analysis, the distance of any two adjacent nodes is assumed to be *r*. For ∀*S*_*i*_ ∈ *S*(*i*=3,…, *n*), *S*_*i*−2_, *S*_*i*−1_, *S*_*i*_, *s* is the neighbor node, where *S*_*i*−2_ is closest to the sink node. *S*_*i*−1_ has two neighbor nodes, *S*_*i*−2_ and *S*_*i*_, defined by *S*_*i*_ as its upstream neighbor node, and *S*_*i*−2_ as its downstream neighbor node.

Suppose that one node has *k*-bits of information to send to another node in the chain. This could be information about temperature, pressure, or salinity, for example. In large-scale wireless sensor networks, data fusion techniques can cut down on the number of packets sent. But in many cases, the data generated by adjacent nodes is often redundant and correlated. However, in underwater networks that use dilute sulfur, more redundant data may not be available, and the data is usually not useful. So, we look at the case where data fusion does not cut down on a lot of data.

First consider the case where each node jumps the packet to the sink node, hereinafter referred to as HBH (Hop by Hop). In this case, the energy expenditure of the nodes in the chain is different. Considering the two adjacent nodes, the *S*_*i*−1_ and the *S*_*i*_, the *S*_*i*−1_ should not only transmit its own data, but also forward the data received from the *S*_*i*_. During the same time, *S*_*i*−1_ transmits more packets than *S*_*i*_, thus resulting in different energy consumption of the nodes. The energy consumption ratio of *S*_*i*−1_ to *S*_*i*_ in each round is *N*. It follows that, under this data transfer mode, the energy near the sink node is depleted earlier.

We again consider the case where each node in the network transfers the data directly to the sin  *k* node, hereinafter referred to as the DIRECT mode. Formulas (2) and (3) show that the energy transmission loss is related to distance in the deep and shallow seas; that is, the farther the sink, the faster the energy exhausted.

Data transmission schemes like the one above show that the unbalanced energy consumption is mostly caused by the different distances between nodes and the different data transmission modes, which use a lot of energy. To solve this problem, we came up with two different ways to balance the amount of energy each node uses and how long the network can last in both the deep and shallow seas.

The article "A Sensor-Based IoT Data Collection and Marine Economy Collaborative Innovation Method" was retracted in 2023. Reasons: unreliable results or conclusions; concerns about the data; concerns about the peer review; concerns about the citations.

## 4. Experiments

This section uses MATLAB to verify the EBH simulation of the energy balance data transfer algorithm. For underwater sensor networks, as for terrestrial wireless sensor networks, they are defined, such as the time period from network operation to the death of the first node in the network or when a certain proportion of the nodes in the network run out of energy and cannot work. Here, the simulations use three survival definitions to evaluate and compare the network survival across the different algorithms.

These three ways are the number of wheels passed from the first network run to the first node in the network, labeled L1, 10% in the network, L10, and 20% in the network, L20.

In addition, the default value of one packet transmission time *T*_TX_ and reception time *T*_RX_ for the node in each round is 40 ms. The transmission time *T*_CX_ of the control information package is 10 ms. We take a received power of 80 mW. For simplicity, in the underwater information monitoring sensor section, we use the sea current velocity sensor with operating power of 200 mW and sampling duration of 50 ms.

For simulation trials, the default operating frequency of the underwater sensor was 25 kHz. The default water depth in shallow waters is 70 m. The default assigned battery energy per node is 2 J. When the node residual energy is less than 2*∗*10^6^ nJ, it is considered out of energy and can no longer work.

There are two graphs on this page: Figures 6 and 7 show how transmission distance and energy use change in shallow and deep water. Both diagrams show that as the distance between nodes increases, so does their electricity use, which means that more energy is used by each of them. The two diagrams also show that the energy consumption of nodes rises as the number of nodes that work at the same time rises. If you are swimming in shallow water, the amount of energy your nodes use will also be influenced by the depth of the water. This is shown in Figure 6. The deeper the sea water, the more the energy the node needs to run. It can also be seen from the diagrams that even though the distance between nodes in shallow water and in deep sea is equal, their energy consumption is greater than that in the deep sea. However, except for the fact that the amount of energy used is different, the energy consumption trend of the two cases is about the same in both cases. For simplicity, only water that is not very deep is shown below. Compared with the traditional method, the method in this paper has lower consumption and can store more energy.

The article "A Sensor-Based IoT Data Collection and Marine Economy Collaborative Innovation Method" was retracted in 2023. Reasons: unreliable results or conclusions; concerns about the data; concerns about the peer review; concerns about the citations.

## 5. Conclusion

Developing the Internet of Things quickly will lead to more changes in the regional economic development model. This will make regional economic growth more efficient, and it will play a bigger role in promoting the long-term development of regional economies. We should pay more attention to the construction and use of the Internet of Things, build a perfect support and service system, promote the deep integration of the Internet of Things and different industries, and play an important role in regional economic development.

Based on the technological determinism, institutional determinism, demand pull theory, and comprehensive dynamic theory of innovation and the relationship and interaction between them, the combination network provides conditions for financial service industry innovation, the opportunity to carry out financial innovation based on the products visually tracked by individuals or enterprises and to establish the dynamic mechanism of financial service industry innovation based on the coordination of technological progress, institution, and demand. On the basis of this theory, this paper makes an empirical analysis on the models of the innovation dynamic mechanism of the financial service industry in the four leading countries of the technological development of the Internet of Things: the United States, Germany, South Korea, and China. Thus, a comparative analysis is made of the development model of the dynamic mechanism of the financial service industry dominated by different factors in different countries. The United States and Germany form a dynamic mechanism of financial service industry innovation driven by demand. South Korea has formed a dynamic mechanism of financial service industry innovation driven by technological progress. China has formed a dynamic mechanism of financial service industry innovation driven by institutional drivers. On the basis of the conclusion of this empirical analysis, combined with the different characteristics of different countries in different stages of economic, technological development and financial system development of the Internet of Things, the conditions and development paths of the dynamic mechanism model dominated by different factors are obtained. First of all, under the three conditions of sufficient supply of IoT technology, marketization, and the potential for large-scale market demand, demand pull as the dominant factor plays an important role here. Small economies (South Korea) under the conditions of imperfect systems but still in line with the overall economic development, and under the conditions of the Internet, take the promotion of technological progress as the leading IoT technology with potential for development; third, large economies (China) with imperfect systems, under the conditions of the demand potential of the Internet of Things and the potential of technological progress, are dominated by institutional reforms.

The article "A Sensor-Based IoT Data Collection and Marine Economy Collaborative Innovation Method" was retracted in 2023. Reasons: unreliable results or conclusions; concerns about the data; concerns about the peer review; concerns about the citations.

## Figures and Tables

**Figure 1:** Three-tier architecture of the Internet of Things.

**Figure 2:** Star network topology.

**Figure 3:** Tree network topology.

**Figure 4:** Network topology.

**Figure 5:** Underwater linear network structure.

**Figure 6:** Energy consumption of underwater sensor networks in the shallow sea.

**Figure 7:** Energy consumption of underwater sensor networks in the deep sea.

**Table 1:** Combination form of Internet of Things industry and traditional industry.

	Combination form	Combined features
Combining the internet of things with the oil and gas sectors	Drilling management: Accurate control of the drilling process, timely early warning pipeline inspection: Improve the automation level of pipeline inspection, reduce human capital investment	Improve the degree of production management in the industry, as well as the safety of the production process and the long-term development of the industry, using InBetter.
The combination of the internet of things and the mining industry	The sensor arrangement in vehicles and miners helmet, in case of an emergency, real-time update equipment and the location of the miners	Improve the safety performance and overall operation efficiency of mining production.
Manufacturing internet of things	Strengthen the management of supply chain	Make supply chain management more predictable, and raise the overall level of product manufacturing quality.
Storage internet of things	Change the traditional inventory management mode and optimize inventory layout	Improving the degree of intelligence in warehouse management and the amount of monitoring in the warehouse environment are two goals.
Smart grid	Intelligent operation and monitoring of power grid	Assist in the overall growth of power grid operation and maintenance, particularly in the area of intelligence.

## Data Availability

The data used to support the findings of this study are available from the author upon request.
